The article "Application of Optimized GA-BPNN Algorithm in English Teaching Quality Evaluation System" was retracted in 2023. Reasons: unreliable results or conclusions; concerns about the data; concerns about the peer review; concerns about the citations.

# Application of Optimized GA-BPNN Algorithm in English Teaching Quality Evaluation System

**DOI:** 10.1155/2021/4123254

**Published:** 2021-12-31

**Authors:** Yaowu Zhu, Junnong Xu, Sihong Zhang

**Affiliations:** ^1^Editorial Office of the Journal, Anhui Vocational College of City Management, Hefei 230011, China; ^2^Institute of Psychology CAS, Beijing 100101, China; ^3^School of Foreign Languages, Hefei Normal University, Hefei 230011, China; ^4^School of Foreign Studies, Hefei University of Technology, Hefei 230011, China

## Abstract

The assessment of teaching quality is a very complex and fuzzy nonlinear process, which involves many factors and variables, so the establishment of the mathematical model is complicated, and the traditional evaluation method of teaching quality is no longer fully competent. In order to evaluate teaching quality effectively and accurately, an optimized GA-BPNN algorithm based on genetic algorithm (GA) and backpropagation neural network (BPNN) is proposed. Firstly, an index system of teaching quality evaluation is established, and a questionnaire is designed according to the index system to collect data. Then, an English teaching quality evaluation system is established by optimizing model parameters. The simulation shows that the average evaluation accuracy of the GA-BPNN algorithm is 98.56%, which is 13.23% and 5.85% higher than those of the BPNN model and the optimized BPNN model, respectively. The comparison results show that the GA-BPNN algorithm in teaching quality evaluation can make reasonable and scientific results.

## 1. Introduction

At present, English is the undisputed world language, which is mainly due to the development of economic globalization. As a bridge tool for communication between different countries, English plays a very important role in international cooperation, information exchange, and technology dissemination. What kind of education belongs to high-quality education? It is essential to assess the teaching quality objectively, find out the problems in teaching in time, and put forward the corrective measures accordingly. Therefore, the same stuff perfect teaching assessment system is a momentous section of teaching work, which can help the education department assess the teaching quality from the aspects of English classroom teaching, teaching achievements, school management, and teachers [1]. In order to improve the problems existing in teaching and improve the teaching quality, it is necessary to clarify the current teaching situation. It is necessary to construct an English teaching quality assessment system suitable for the actual situation of universities. The self-positioning of universities determines that the assessment of teachers' teaching quality not only can be assessed by theoretical teaching but also can pay close attention to the development of students' practical skills so that students have a solid theoretical foundation and practical ability that satisfy the demand of social development. Therefore, the assessment of teaching quality is a significant content of teaching management [2, 3].

The assessment of teaching quality in universities is a fuzzy and complex nonlinear question, which is mainly manifested in a wide range of assessment contents and a large number of indicators. Researchers use grey relational analysis, analytic hierarchy process, and fuzzy all-round assessment to assess teaching quality [4–6]. Although various assessment factors are fully considered, it is difficult to eliminate subjectivity and randomness, which has certain limitations on nonlinear teaching quality assessment. With the successive expansion of computer, Internet, and artificial intelligence, new means, for example, BP neural network (BPNN), have appeared in the research of teaching quality assessment [7]. BPNN, which is suitable for dealing with nonlinear problems and has a self-learning function, can ameliorate the exact of teaching quality assessment to a certain extent. However, because the descent learning method adopted by neural network is local search, it is simple for neural network to divide into local minimum, and its generalization ability is weak. In view of these shortcomings, literature [8] selects the maximum entropy criterion with the function of describing uncertainty distribution information to replace the mean-square-error criterion of BP algorithm and establishes the maximum entropy neural network assessment model of teaching quality. The relative error of the improved model is relatively small, and the results show that the method has certain generalization ability and credibility. Literature [9] uses PSO neural network technology to establish a teaching quality assessment system in universities. The system takes teaching assessment criteria as input and teaching assessment results as output. The assessment outcome shows that this means may better put up with the weak point of conventional teaching quality assessment means.

With the introduction of neural network in teaching quality assessment in recent years, the shortcomings based on a traditional prediction model have been greatly overcome, and the results are good [10]. Nevertheless, because the ordinary neural network algorithm is easy to be limited to the minimum locally, it cannot improve the convergence speed, so it is difficult to make the learning results of the network converge accurately.

In this paper, we have concluded some contributions as follows: (1) the GA-BPNN model is proposed and applied to study the English teaching quality evaluation model; (2) compared to other baseline methods, the simulation shows that the average evaluation accuracy of the GA-BPNN model is 98.56%, which is 13.23% and 5.85% higher than the BPNN model and the optimized BPNN model, respectively; and (3) results show that the GA-BPNN model in teaching quality evaluation can make reasonable and scientific results.

In this paper, the work is composed of six sections. In the first section, we analyzed the background in English teaching quality evaluation and summarized the contributions. In the second section, we discussed some related papers and their contributions in this area. In the third section, we proposed the GA-BPNN model and presented its theories. In the fourth section, we constructed the English teaching quality evaluation system. In the fifth section, we discussed the computed results by the designed system and also compared the proposed system to other baseline methods. In the sixth section, we concluded this work and presented the limitations.

### 1.1. Related Work

The assessment of college English teaching quality is a complex problem. English teaching includes many factors such as teaching conditions, course difficulty, teachers' teaching, and learning effect, which interact with each other. At the same time, the relationship between teachers and students is complex, and there are many factors. At present, there is no recognized and ideal assessment system of English classroom teaching quality. Literature [11] thinks that the standard of measuring teaching quality should not be school reputation but should be carried out around various indicators that affect students' mental development. Literature [12] divides the assessment of education quality into four dimensions, which are background, development, internal consistency, and external consistency. Literature [13] advocates that the assessment of teaching quality should be carried out from three dimensions, namely the quality in classroom concept, the quality in economic concept, and the quality in value judgment. Literature [14, 15] analyze the basic characteristics of China's primary and secondary education assessment from three aspects: structure, function, and social function and point out that there are some problems in China's education assessment, such as utilitarian tendency, single education assessment standard, lagging education assessment system, and rigid system. Literature [16] advocates that education reform should be combined with assessment reform, and education quality assessment reform cannot be analyzed in isolation. Literature [17] holds that it is necessary to innovate the system of teaching quality assessment under the direction of the scientific conception of burgeon, seek reform in innovation, and promote progress in reform. Literature [18] holds that the improvement of education quality depends on the innovation of the teaching system, and the teaching system should be changed with the development of society.

At present, scholars have done research on teaching quality assessment models for different school types, different disciplines, and different majors. Literature [19] has designed the teaching quality assurance system for undergraduate students in research universities, extracted the important factors affecting the assessment of teaching quality, and put forward the implementation countermeasures for the key factors, thus providing a more reasonable and effective system for the assurance of teaching quality. Literature [20] is a research on the construction of a practical teaching system in application-oriented universities. Through empirical research, it provides reliable theoretical support for the cultivation of applied talents and the assessment of teaching quality in practice-oriented universities. Literature [21] combines the characteristics of military school teaching and the requirements of the Ministry of Education for military school education and establishes a military school teaching quality assessment system in view of BPNN so as to realize scientific, reasonable, and timely assessment of military school teaching quality. Literature [22] uses fuzzy comprehensive assessment means to assess the teaching quality of MOOC in college physics from three aspects: the degree of achieving teaching objectives, the rationality of teaching content, and the conformity of teaching assessment and feedback. Based on the assessment results, the existing problems in MOOC English classroom teaching of college physics are analyzed.

## 2. Methods

The research history of the genetic algorithm (GA) is correspondingly shorter. Starting with trying to expound the complex adaptation process of organisms in natural systems, the artificial system pattern was built by simulating the mechanism of biological evolution.

Resident is made up of a certain quantity of personal code by genes. Each personal code is in fact a substance with chromosome characteristics. As the major germ carrier of genetic makings, a chromosome is a gathering of polygenes, and its inner indicate (expression gene) is determined by some integration of genes. Therefore, the mapping from phenotype to genotype, that is, coding, needs to be realized at the beginning. This procedure will bring about the offspring resident whose population is like natural evolution adapting to the circumstances more than the former produce, and the best individual in the final produce resident can be translated as the close to the best solution of the question.

The neuron structure diagram is shown in Figure 1, in which purple tentacles gather around the cell body. Dendrites receive external stimuli and transmit stimulation signals into the nucleus for information processing, which is the input of information. In the picture, yellow pith, Schwann cells and cell knots are used to connect two neurons, namely axons. The main function of the axon is to transmit the information of one neuron to other neurons, which is the output of neurons. The human brain is composed of 86 billion such neurons, and all thinking consciousness is realized by connecting them into a network.

BPNN is a multilayer feedforward network with mistaken back spread [23–25]. The composition of BPNN can be simplified as nodes and arrows. Nodes imitate dendrites to receive input information, and arrowheads imitate axons of neurons to transmit information channels. According to the distribution of neurons, neural networks can be divided into input layer, hidden layer, and output layer. There is no connection between nodes in the same layer, and nodes in different layers are connected according to the arrow direction. Data is input through the nodes of the input layer, and the nodes of the hidden layer and the output layer activate and operate the data.

Activation is the process of mathematically deforming the values obtained by summing nodes. For example, Figure 2 is the structure diagram of BPNN, which can be expressed as *y*_1_=*g*(*x*_1_).

The essence of the BPNN model algorithm is to constantly adjust the network model parameters by propagating the calculation errors backward and correcting the errors at the same time so as to keep close to the one-to-one correspondence of targets. Therefore, the neural network model can be optimized by using the training set to train it. The convergence of the training process is analyzed to determine whether it converges and whether its convergence performance is good or bad. Through the test data set, the accuracy and practicability of the predicted value are verified.

The neural network algorithm is simple to separate into local minima, slow in aggregate, and poor in global searching ability, while the GA not only has continuity of an objective function but also has the good global searching ability, and it is easy to get worldwide the best solution or suboptimal solution with better performance. Therefore, the combination of GA and BPNN algorithms can achieve the effect of complementary advantages.

The implementation process is to optimize the weights and thresholds of network connection by GA, train by BP learning algorithm, and verify the test samples by using the generalization capacity of neural network. The steps are as follows [26, 27]:

(1) The BPNN is established, and the teaching performance indicators in the training sample set are given as the input and *T* as the output vector.
(2) A group of *P* individuals are randomly generated; each individual represents the initial weight-threshold distribution of a neural network; and the length of the individual is the sum of the number of individuals and the threshold number of neural network weights, namely
  (1) $$\begin{array}{c} n=r*s_{1}+s_{1}*s_{2}+s_{1}+s_{2}, \end{array}$$
where *n* is the coding length of GA, *s*_1_ is the quantum of hidden layer nodes, *s*_2_ is the length of the output vector, and *r* is the length of the input vector.
(3) Design a fitness function associated with the error function, where the fitness function
  (2) $$\begin{array}{c} f=\frac{1}{E+1},E=\frac{1}{2}\sum_{k=1}^{n}{\left(d_{k}-o_{k}\right)}^{2}, \end{array}$$
where *d*_*k*_ and *o*_*k*_ are the expected output and actual output of *k* groups of data, and the personal is appraised according to the healthy effect value.
(4) Choose the chromosome with strong adaptability, keep the current optimal solution in each generation of inheritance, and enter the next generation directly until it meets the precision requirement or the maximum algebra of 100. At this time, select, cross, and mutate the chromosome according to the law to produce the next generation population.
(5) Repeat steps (3) and (4) and obtain the individual with the largest fitness as the primary value and threshold value of BPNN after repeated iteration.
(6) Backpropagation of information and error is used to train BPNN so that the error converges to the specified precision range.
(7) After the above calculation steps, the BPNN after training is used to assess the assessment samples.

The specific flow of the GA-BPNN combination model is shown in Figure 3.

### 2.1. English Teaching Quality Evaluation

Teaching quality assessment involves many factors. The index system of this paper is established by referring to the opinions of frontline teachers, teaching experts, and teaching quality assessment management departments, consulting literature and drawing lessons from the teaching quality assessment index system of some universities. The assessment index system of teaching quality is divided into 5 first-class indexes and 18 second-class indexes, which are numbered *X*_1_ ~ *X*_18_, as shown in Table 1.

As the output of the neural network, the assessment results of teachers' teaching quality are separated into five ranks: excellent, good, fair, passing, and failing. The output range of each rank is shown in Table 2.

### 2.2. Data Collection and Processing

According to the content of the index system, the questionnaire was designed, 100 questionnaires were distributed, 90 were recovered, and 92 valid questionnaires were screened, that is, 92 valid data groups. The transmission function used in the output layer of the neural network is a shape function, and its value range is [0, 1], that is, the output range of the neural network is [0, 1], so the output of training data should be normalized to [0, 1]. The scoring data should be standardized to [0, 1]. The max-min method, a common normalization method, can well preserve the original meaning of the data, so this method is used to normalize the data.

The calculation of this method is shown in the following formula:

(3) $$\begin{array}{c} X=\frac{I-I_{\min}}{I_{\max}-I_{\min}}, \end{array}$$

where *X* is the normalized score, i.e., BPNN input value, *I*_min_ is the minimum score of teaching quality, *I*_max_ is the maximum score, and *I* is the untreated score.

The processed sample data of some students' assessment are shown in Table 3.

### 2.3. Structure Design of BPNN Model

The procedure of building up the BPNN model is as follows: firstly, establish the neural network construction, that is, determine the quantum of input nodes, output nodes, hidden layers, and nodes in each layer. Adjust the structure of the BP network and building up the primary network factor, and the practice and learning of the neural network begin. When the network tends to be stable after acquiring knowledge, the actual output reaches the specified error requirements or the number of repeated training reaches the specified maximum, and the training ends. At the same time, the test data set is used to evaluate the trained neural network. If it reaches the specified accuracy, the BPNN model has deterministic significance [28–30].

The assessment indexes of students' assessment of teaching are separated into four first-class indexes, 12 second-class indexes, and the 12 second-class assessment indexes that are adopted as the inputs of the input layer of the neural network. Therefore, the number of nodes in the input layer of BPNN is 12 accordingly. Because there is only one result of students' teaching assessment, the output layer of the network is only set as one output node. The value limits are [0, 1].

At present, a common method to determine the best quantity of hidden layer nodes is test and mistaken means [31–34]. When using test and mistaken means, some empirical expression to determine the quantity of hidden layer nodes may be adopted. The common ones are [27] as follows:

(4) $$\begin{array}{c} m=\sqrt{n+l}+a, \end{array}$$

(5) $$\begin{array}{c} m=\;\log_{2}\;n, \end{array}$$

(6) $$\begin{array}{c} m=\sqrt{nl}. \end{array}$$

where *m* is the quantity of hidden layer nodes, *n* is the quantity of input layer nodes, 1 is the quantity of output layer nodes, and *a* is a constant between 1 and 10. In the light of formula (4), the number of hidden layer nodes is 5–14, and the best quantity of hidden layer nodes is 7.

The Tansig hyperbolic tangent function is selected as the activation function on the hidden layer unit. In the training data specimen set, the prevenient output values of the assessment results all fall within the space of [0, 1] after normalization, so the sensitization functions on the output layer units are all taken as Sigmoid functions, and the effect forms are as follows:

(7) $$\begin{array}{c} f\left(x\right)=\frac{1}{1+e^{-x}}. \end{array}$$

In this network construction, the input vector is *X*=(*x*_1_, *x*_2_,…,*x*_12_)^*T*^, and the weight from the input layer unit *i*to the hidden layer unit *h* is *W*=(*w*_11_, *w*_12_,…, *w*_12,7_).

The output of hidden layer is *Y*=(*y*_1_, *y*_2_,…, *y*_7_), and the weight from hidden layer to output layer is *W*=(*w*_1_, *w*_2_,…, *w*_7_);

The actual output of the network is *O*=net(*Y*), and *T*=(*t*) indicates the prevenient output of the training specimen. The output of hidden layer node *h* and output of output layer node *s* are as follows:

(8) $$\begin{array}{c} y_{h}^{k}=f\left(\sum_{i=1}^{12}w_{ih}x_{i}^{k}+\theta_{h}\right),\\ o_{h}^{k}=g\left(\sum_{h=1}^{7}w_{h}y_{h}^{k}+\theta \right). \end{array}$$

## 3. Results and Analysis

### 3.1. The Result of GA-BPNN Model

In order to verify the performance of this model, the BP neural network method is used to simulate the sample data, and a comparative experiment is carried out. The simulation experiment of English teaching quality assessment is realized by MATLAB programming, and the mean-square-error variation diagram of BPNN optimized by GA is shown in Figure 4.

Figure 4 shows that the BPNN model optimizing by GA meets the stopping condition in the 60th generation, that is, the number of convergence steps is 60, which indicates that the BPNN model optimizing by GA can accelerate the convergence speed of the network.

The prediction accuracy percentage is shown in Figure 5.

It can get from Figure 5 that the forecast accuracy percentage of 29 groups of 30 test samples is above 97%, and the prediction accuracy of 22 groups is above 98%. It can be seen that the GA-BPNN model has a good approximation effect.

The sum of squares of GA-BPNN errors is shown in Figure 6.

Figure 6 shows that the sum of squares of errors converges quickly before the 6th generation, while the convergence speed of the 10th–30th generation is relatively slow. After the iteration number is 35th generation, the sum of squares of errors of the network is stable, indicating that the GA-BPNN model can achieve global optimization quickly. It can be seen that the model has high adaptability.

The fitness function curve of GA-BPNN is shown in Figure 7.

Figure 7 shows that the training fitness function of GA-BPNN converges quickly before the 10th generation and basically reaches a stable state after 43 iterations. It can be seen that the model has high adaptability. In a word, the internal mechanism of GA-BPNN determines its training and prediction performance. Considering the prediction accuracy and adaptability, the GA-BPNN English teaching quality assessment model is effective and robust. Individual samples of the BPNN model have a large deviation from the pretest results, and the prediction results of the GA-BPNN model are stable. Compared with the BPNN teaching quality evaluation model, it can be seen that the GA-BPNN evaluation model has better performance. The evaluation accuracy of the improved model is obviously higher than that of the BP neural network model that is optimized by genetic algorithm. Therefore, the BP neural network evaluation model based on the improved genetic algorithm has better application value, and the model can make a timely, effective, and scientific evaluation of teaching quality.

### 3.2. Model Comparison

The contrast outcomes of average assessment precise are shown in Figure 8. The average assessment accuracy of the BPNN model for 100 groups of data is 85.33%, the average assessment accuracy of the traditional optimized BPNN model is 92.71%, and the average assessment accuracy of the GA-BPNN algorithm is 98.56%, which is 13.23% and 5.85% higher than the two methods, respectively. It can be seen that the GA-BPNN algorithm has better assessment results. The comparison results show that the BP neural network teaching quality evaluation model optimized by a genetic algorithm based on adaptive mutation can make reasonable and scientific evaluation results on teaching quality.

The weights of the BP neural network trained by GA can get satisfactory results. However, because the improved algorithm will perform genetic operations such as coding, decoding, crossover, and mutation on a large number of data, the running time is longer than that of an ordinary BP algorithm.

## 4. Conclusions

The evaluation of teaching quality is a very complex and fuzzy nonlinear process, which involves many factors and variables, so the establishment of the mathematical model is complicated, and the traditional evaluation method of teaching quality is no longer fully competent. The GA-BPNN algorithm constructed in this paper is obviously superior to the prediction results of a pure neural network in training speed and fitting results. The reason is that the effect and performance of the traditional neural network model are greatly limited by the random initialization of weights and thresholds, and the convergence effect of the network is not ideal. The GA-BPNN algorithm constructed in this paper searches locally near the global optimal solution, which can well overcome the problem of slow convergence speed of the traditional algorithm and, at the same time, overcome the problem that it is easy to be locally limited to the minimum. The neural network is used to assess the English classroom teaching quality reasonably, which put up with the immediate effect of mankind element on the assessment outcome. It develops a new means to reasonably evaluate the quality of English classroom teaching and provides a meaningful reference value for the research of English teaching quality evaluation. However, this paper does not evaluate the stability of the Internet in the quality of English classroom teaching. In future work, more data need to be collected for demonstration.

## Figures and Tables

**Figure 1:** Neuron structure diagram.

**Figure 2:** Structure diagram of BPNN.

**Figure 3:** Algorithm flowchart of GA-BPNN combination model.

**Figure 4:** GA-BPNN mean square error.

**Figure 5:** GA-BPNN prediction accuracy percentage.

**Figure 6:** Sum of squares of GA-BPNN errors.

**Figure 7:** GA-BPNN fitness function curve.

**Figure 8:** Comparison of model performance.

**Table 1:** Assessment index system of English teaching quality.

First-class assessment index	Secondary assessment index	Indicator code
Teachers' quality	Clear educational objectives	*X*_1_
	Solid professional knowledge	*X*_2_
	Teaching and explaining level	*X*_3_

Teaching attitude	Counseling and answering questions are patient and positive	*X*_4_
	Teaching is serious and infectious	*X*_5_
	Strict attitude and excellence	*X*_6_

Content of courses	The conceptual theory is accurate	*X*_7_
	Full of content and attention to ability	*X*_8_
	Connect with practice and pay attention to practice	*X*_9_
	Depth and breadth of professional knowledge	*X*_10_

Teaching method	Be good at enlightening and guiding thinking	*X*_11_
	Various ways and proper application	*X*_12_
	Pay close attention to individuality and teach students in agreement with their ability	*X*_13_
	Focus on stimulating innovation consciousness	*X*_14_

Teaching effect	Self-study ability and interest in learning have improved	*X*_15_
	Understanding and mastering the basic knowledge	*X*_16_
	Ameliorate the ability to analyze and solve problems	*X*_17_
	Comprehensive quality and innovative ability	*X*_18_

**Table 2:** Grades of assessment results and their output ranges.

Rank	Excellent	Good	Medium	Get through	Failing
Output range	[0.9, 1]	[0.8, 0.89]	[0.7, 0.79]	[0.6, 0.69]	[0, 0.59]

**Table 3:** Sample data of student assessment.

Indicator code	Sample serial number					Assessment results
	1	2	3	4	…	
*X*_1_	0.88	0.88	0.74	0.86	…	0.88
*X*_2_	0.83	0.75	0.92	0.74	…	0.78
*X*_3_	0.96	0.96	0.86	0.93	…	0.93
*X*_4_	0.87	0.94	0.80	0.58	…	0.91
*X*_5_	0.91	0.82	0.91	0.64	…	0.96
*X*_6_	0.93	0.84	0.76	0.78	…	0.76
*X*_7_	0.86	0.88	0.55	0.90	…	0.88
*X*_8_	0.77	0.97	0.63	0.88	…	0.89
*X*_9_	0.83	0.91	0.79	0.96	…	0.95
*X*_10_	0.94	0.80	0.91	0.43	…	0.91
*X*_11_	0.97	0.71	0.87	0.69	…	0.77
*X*_12_	0.91	0.83	0.66	0.71	…	0.83
*X*_13_	0.87	0.91	0.59	0.55	…	0.81
*X*_14_	0.81	0.88	0.77	0.96	…	0.90
*X*_15_	0.66	0.56	0.43	0.92	…	0.88
*X*_16_	0.91	0.74	0.58	0.68	…	0.92
*X*_17_	0.81	0.83	0.91	0.75	…	0.91
*X*_18_	0.73	0.91	0.71	0.61	…	0.85

## Data Availability

The data used to support the findings of this study are available from the corresponding author upon request.

## References

[1] Ait Hammou B., Ait Lahcen A., Mouline S. (2020). Towards a real-time processing framework based on improved distributed recurrent neural network variants with fastText for social big data analytics. *Information Processing & Management*.

[2] Guo M., Xiong X., Feng G. (2019). A research on behavioral deviation and reform program of teaching quality assess in experiment and training of colleges. *Research and Exploration in Laboratory*.

[3] Yao Y., Wang J., Long P., Xie M., Wang J. (2020). Small‐batch‐size convolutional neural network based fault diagnosis system for nuclear energy production safety with big‐data environment. *International Journal of Energy Research*.

[4] Lu Y., Cen Y. T. (2017). Research of community education curriculum teaching quality assess model base on two-tuple linguistics. *Mathematics in Practice and Theory*.

[5] Ye J. (2017). On the construction of teaching quality assessment system in universities. *Education Forum*.

[6] Parwez M. S., Rawat D. B., Garuba M. (2017). Big data analytics for user-activity analysis and user-anomaly detection in mobile wireless network. *IEEE Transactions on Industrial Informatics*.

[7] Esteban C. M. R., del Cerro J. S. (2020). Teaching quality: the satisfaction of university students with their professors. *Anales de Psicología/Annals of Psychology*.

[8] Song W., Xu Y., Li G. H. (2018). English teaching quality assess of computer major under the background of international talent training. *Education Modernization*.

[9] Zhang X. H. (2018). Comments on teaching quality assess of universities teachers. *Modern Vocational Education*.

[10] Liu Y. Research on teaching reform of rehabilitation nursing major based on modern apprenticeship system. *Frontiers of Nursing*.

[11] Li J., Li X. W. (2017). Application of pdca management mode in teaching quality assess of clinical teaching in ct room. *China Continuing Medical Education*.

[12] Zhu Y. (2019). Construction of mixed teaching mode and quality assessment system for mechan-ical design courses in applied universities. *China Modern Educational Equipment*.

[13] Nie J., Zhou P. Physical optics teaching design under the mode of CDIO education.

[14] Xu S., Connelly F. M. (2009). Narrative inquiry for teacher education and development: focus on English as a foreign language in China. *Teaching and Teacher Education*.

[15] Zhang F., Liu Y. (2014). A study of secondary school English teachers’ beliefs in the context of curriculum reform in China. *Language Teaching Research*.

[16] Dang D. C., Eremeev A., Lehre P. K. Non-elitist evolutionary algorithms excel in fitness landscapes with sparse deceptive regions and dense valleys.

[17] Das S. P., Padhy S. (2018). A novel hybrid model using teaching-learning-based optimization and a support vector machine for commodity futures index forecasting. *International Journal of Machine Learning and Cybernetics*.

[18] Khoshnoudi-Nia S., Moosavi-Nasab M. (2019). Prediction of various freshness indicators in fish fillets by one multispectral imaging system. *Scientific Reports*.

[19] Zhang R., Meng F., Zhou Y., Liu B. (2018). Relation classification via recurrent neural network with attention and tensor layers. *Big Data Mining and Analytics*.

[20] Huang P., Chris R., Craig R. (2018). Satellite selection with an end-to-end deep learning network. *GPS Solutions*.

[21] Krizhevsky A., Sutskever I., Hinton G. E. (2017). ImageNet classification with deep convolutional neural networks. *Communications of the ACM*.

[22] Hassib E. M., El-Desouky A. I., Labib L. M., El-kenawy E.-S. M. (2020). WOA + BRNN: an imbalanced big data classification framework using Whale optimization and deep neural network. *Soft Computing*.

[23] Kumari N., Kr Bhatt A., Kr Dwivedi R., Belwal R. (2021). Hybridized approach of image segmentation in classification of fruit mango using BPNN and discriminant analyzer. *Multimedia Tools and Applications*.

[24] Rostami A., Anbaz M. A., Erfani Gahrooei H. R., Arabloo M., Bahadori A. (2018). Accurate estimation of CO_2_ adsorption on activated carbon with multi-layer feed-forward neural network (MLFNN) algorithm. *Egyptian Journal of Petroleum*.

[25] Gong C., Xu D., Zhou Z., Vitiello N., Wang Q. (2020). BPNN-based real-time recognition of locomotion modes for an active pelvis orthosis with different assistive strategies. *International Journal of Humanoid Robotics*.

[26] Shamsolmoali P., Zareapoor M., Yang J. (2019). Convolutional neural network in network (CNNiN): hyperspectral image classification and dimensionality reduction. *IET Image Processing*.

[27] Mohan B. P., Khan S. R., Mba L. (2020). High pooled performance of convolutional neural networks in computer-aided diagnosis of gi ulcers and/or hemorrhage on wireless capsule endoscopy images: a systematic review and meta-analysis. *Gastrointestinal Endoscopy*.

[28] Lee K. Y., Kim K. H., Kang J. J. (2017). Comparison and analysis of linear regression & artificial neural network. *International Journal of Applied Engineering Research*.

[29] Ghosh S., Chattopadhyay B. P., Roy R. M., Mukherjee J., Mahadevappa M. (2019). Estimation of echocardiogram parameters with the aid of impedance cardiography and artificial neural networks. *Artificial Intelligence in Medicine*.

[30] Pan F., Wen H., Gao X., Pu H., Pang Z. (2020). Clone detection based on BPNN and physical layer reputation for industrial wireless CPS. *IEEE Transactions on Industrial Informatics*.

[31] Zhang P., Cui Z., Wang Y., Ding S. (2021). Application of BPNN optimized by chaotic adaptive gravity search and particle swarm optimization algorithms for fault diagnosis of electrical machine drive system. *Electrical Engineering*.

[32] Samantaray S., Sahoo A. (2020). Prediction of runoff using BPNN, FFBPNN, CFBPNN algorithm in arid watershed: a case study. *International Journal of Knowledge-Based and Intelligent Engineering Systems*.

[33] Sayahi T., Tatar A., Rostami A., Anbaz M. A., Shahbazi K. (2021). Determining solubility of CO_2_ in aqueous brine systems via hybrid smart strategies. *International Journal of Computer Applications in Technology*.

[34] Hairuddin N. L., Yusuf L. M., Othman M. S., Nasien D. (2021). Gender classification using a PSO-based feature selection and optimised BPNN in forensic anthropology. *International Journal of Computer Aided Engineering and Technology*.

